# Carbon Monoxide-Releasing Molecule-3 Suppresses the Malignant Biological Behavior of Tongue Squamous Cell Carcinoma via Regulating Keap1/Nrf2/HO-1 Signaling Pathway

**DOI:** 10.1155/2022/9418332

**Published:** 2022-09-16

**Authors:** Yan Dai, Hui Chen, Yan Pan, Hui Song

**Affiliations:** ^1^Department of VIP Center, School and Hospital of Stomatology, Cheeloo College of Medicine, Shandong University, No. 44-1 Wenhua Road West, 250012 Jinan, China; ^2^Department of Oral and Maxillofacial Surgery, Zibo Central Hospital, 54 West Gongqingtuan Road, 255036 Zibo, China; ^3^Department of Endodontics, Jinan Stomatology Hospital, No. 101 Jingliu Road, 250001 Jinan, China; ^4^Department of Geriatric Stomatology, Yantai Stomatology Hospital, No. 142 Beida Street, 264008 Yantai, China; ^5^Shandong Key Laboratory of Oral Tissue Regeneration & Shandong Engineering Laboratory for Dental Materials and Oral Tissue Regeneration, No. 44-1 Wenhua Road West, 250012 Jinan, China

## Abstract

Carbon monoxide-releasing molecule-3 (CORM-3) is a water-soluble complex which has the ability to release carbon monoxide (CO). The study is aimed at investigating the epidemiological characters and effects of CORM-3 on tongue squamous cell carcinoma (TSCC) cells and the mechanisms involved. Firstly, CAL27 and SCC4 were treated with CORM-3 or iCORM-3. The proliferation, migration, and invasion of cells were separately evaluated by CCK-8, scratch assay, and transwell assay. We found that the optimal concentration of CORM-3 on the proliferation of CAL27 and SCC4 cells was 400 *μ*M, and CORM-3 was significantly inhibited the proliferation, migration, and invasion of TSCC cells. Meanwhile, CORM-3 increased the protein expression of HO-1 detected by western blot. Short-hairpin RNAs (shRNAs) were constructed to manipulate the expression of HO-1 in CAL27 and SCC4 cells. Then, rescue assays were conducted to explore the reversion effect of shHO-1 on the CORM-3 function. Mechanistically, CORM-3 decreased the protein of Keap1 expression as well as increased Nrf2 expression. Upregulation of E-cadherin was observed, as well as the downregulation of N-cadherin expression significantly. The antitumor effect of CORM-3 was used to xenograft tumor in nude mice for further investigation *in viv*o, and the result showed that CORM-3 significantly suppressed tumor growth in xenograft nude mice. These data suggest that CORM-3 acts as a tumor suppressor by regulating the Keap1/Nrf2/HO-1 signaling pathway in TSCC, which provides a potential chemotherapeutic strategy for TSCC.

## 1. Introduction

TSCC is the most common type of head and neck squamous cell carcinoma (HNSCC) and is known for its ability of proliferation and high metastasis [1]. It is characterized by high invasiveness and early lymphatic metastasis to adjacent tissues and organs because the tongue has many lymphatic vessels and abundant blood circulation [2]. Although TSCC treatments are constantly improving with the advancement of technology, the mortality rate is still high [3]. Therefore, it is important to identify possible molecular pathways relevant to the progression of TSCC and to find novel therapeutic strategies.

CO is a by-product of heme oxygenase catalyzed by heme production and is considered as a toxic gas for a long time. However, recent studies suggested that CO has cytoprotective effects such as vasodilation, inhibition of cell apoptosis, inhibition of inflammation, and protection of organ ischemia-reperfusion injury [4, 5]. CORMs are newly synthesized CO compounds that can effectively release controlled amounts of CO in biological models *in vivo* and *in vitro* under appropriate conditions [6]. In particular, CORM-3 is completely water-soluble and can release CO quickly when dissolved in a physiological solution [7]. Previous studies have shown that CORM-3 inhibits the expression of inflammatory factors and reduces the infiltration and adhesion of immunocompetent cells by releasing CO [8]. Besides, it has been confirmed that CORM-3 could prevent the recurrence of sepsis and have antitumor effect on breast cancer [9].

Nrf2 gene plays an important role in tumor cells [10–12]. It can induce the expression of a complex network of nearly 500 genes, which encode proteins with different antioxidant and cytoprotective functions [13]. Heme oxygenase 1 (HO-1) is an important downstream target gene of Nrf2 [14]. It has powerful antioxidant and antiapoptotic effects and has an important regulatory effect on cancer cell growth and treatment resistance. It is reported that HO-1 has a certain inhibitory effect on prostate cancer, which may be attributed to its regulatory effect on proangiogenic factors by significantly downregulating VEGF-A, VEGF-C, and MMP-9 expression level [15] and inhibiting the NF-*κ*B signaling pathway [16]. In addition, overexpression of HO-1 can also significantly inhibit cell proliferation, migration, and angiogenesis potential and inhibits tumor cell growth in non-small-cell lung cancer cells [17]. Under physiological conditions, CORM-3 can increase the expression of HO-1 in various animal models and cell types [18, 19]. Therefore, we hypothesized that CORM-3-released CO, which in turn induces the expression of HO-1, plays a biological role in the tumor microenvironment through the Nrf2/HO-1 signaling pathway.

Despite many beneficial effects of CORMs that have been proven, the effects of CORM-3 on TSCC and related molecular mechanisms are still unclear. The present study is aimed at evaluating the effects of CORM-3 in two different TSCC cell lines *in vivo* and *in vitro* and at exploring the possible molecular mechanism.

## 2. Materials and Methods

### 2.1. Reagents and Antibodies

CORM-3 was purchased from Sigma Japan Inc. (Tokyo, Japan). CORM-3 solution was prepared by dissolving the compound in distilled water when it is in need. Meanwhile, iCORM-3 is prepared by dissolving CORM-3 in a phosphate buffer and standing to release CO at room temperature for 48 hours. Eliminate residual CO by bubbling the previous solution with N_2_ [20]. The following reagents were purchased from designated sources: anti-E-cadherin rabbit polyclonal antibody (cat no. 20874-1-AP), anti-N-cadherin rabbit polyclonal antibody (cat no. 22018-1-AP), anti-Keap-1 rabbit polyclonal antibody (cat no. 10503-2-AP), and anti-Nrf2 rabbit polyclonal antibody (cat no. 16396-1-AP) were purchased from Proteintech Group, Inc. (Chicago, IL, USA). Anti-HO-1 rabbit polyclonal antibody (cat no. ab13243) was the product of Abcam (Cambridge, MA, USA). Anti-GAPDH rabbit monoclonal antibody, anti-rabbit IgG secondary antibody, and anti-Ki67 rabbit monoclonal antibody were from Cell Signaling Technology (Beverly, USA).

### 2.2. CAL27 and SCC4 Cell Culture and Treatment

Human TSCC cell lines CAL27 and SSC4 were obtained from the Chinese Academy of Sciences Committee Type Culture Collection Cell Bank (Shanghai, China). CAL27 cells were cultured in H-DMEM (Gibco, Grand Island, NY, USA) supplemented with 10% fetal bovine serum (FBS) and penicillin/streptomycin (Gibco, Grand Island, NY, USA). SCC4 cells were cultured in DMEM/F-12 (Gibco, Grand Island, NY, USA) supplemented with 10% FBS and penicillin/streptomycin (Gibco, Grand Island, NY, USA). The cells were cultured in an incubator at 37°C, 5% CO_2_, and saturated humidity. When the cell fusion reaches 70-80%, the cells were digested with 0.25% trypsin and subcultured. In subsequent experiments, CAL27 and SCC4 cells were treated with 0, 100, 200, 400, and 800 *μ*M CORM-3 for 24 h or with 0, 200, 400, and 800 *μ*M CORM-3 for 0 h, 6 h, 12 h, 24 h, 48 h, and 72 h, respectively, *in vitro*.

### 2.3. Cell Proliferation Assay

Cell Counting Kit-8 (CCK-8; Dojindo Molecular Technologies, Inc., Beijing, China) assay was performed to check the cell proliferation. CAL27 and SCC4 cells were inoculated in 96-well plates (1000 cells/well) and cultured in complete medium (DMEM and DMEM/F-12 supplemented with 10% FBS) containing different concentrations of 0, 100, 200, 400, and 800 *μ*M CORM-3for 24 h. The cells were also treated with 0, 200, 400, and 800 *μ*M CORM-3 for 0 h, 6 h, 12 h, 24 h, 48 h, and 72 h. Subsequently, 10% CCK-8 solution was added to each well at 37°C for 2 h. The optical density (OD) absorbance was measured at 450 nm using a microplate reader (Spectro Analytical Instruments GmbH, Kleve, Germany). The assay was done in triplicate, and each experiment was repeated three times.

### 2.4. Cell Migration

Cell migration was measured using the scratch assay. The exponentially growing CAL27 or SCC4 cells were trypsinized and resuspended to the density of 5 × 10^4^/ml, respectively. The cells were then seeded into 6-well cell culture plates. When the cells reach 80% confluence, the scratch was created using a disposable sterile 200 *μ*l pipette tip. After injury, the cells were gently washed with PBS and cultured in serum-free medium (control group), 400 *μ*M CORM-3 (CORM-3 treatment group), and 400 *μ*M iCORM-3 (iCORM-3 treatment group). The injured monolayer was examined and photographed at 0 h, 6 h, 12 h, and 24 h after scratching, and migration was evaluated using Image-Pro Plus 6.0 measurement software.

### 2.5. Cell Invasion

Cell invasion experiments were performed using Corning Matrigel Invasion Chamber (Corning Co, Corning, USA). A concentration of 200 *μ*l CAL27 or SCC4 cell suspension of 4 × 10^5^/ml was separately added to the upper chamber, respectively, while 600 *μ*l of 10% FBS-DMEM was added to the lower chamber. After 24 hours of incubation in a 5% CO_2_ incubator at 37°C, the noninvading cells were removed with a cotton swab. The lower surface of the invaded cells was fixed in 4% paraformaldehyde for 15 minutes and stained with 0.1% crystal violet for 15 minutes. The cell invasion value was determined by counting the stained cells with an optical microscope (×100). The experiment was repeated three times.

### 2.6. Western Blotting Assay

To further investigate the effect of CORM-3 on the expression of HO-1 protein in CAL27 and SCC4 cells, western blot analysis was used to detect the expression of HO-1 during CORM-3(0, 100, 200, and 400 *μ*M) stimulation for 24 h. In order to explore the potentially related signaling molecules, CAL27 and SCC4 cells were stimulated by CORM-3 (400 *μ*M) for different time (0, 0.25, 0.5, 1, 3, 6, and 12 h).

The total protein was extracted from cells using RIPA buffer (Beyotime Institute of Biotechnology, Jiangsu, China). Equal amounts of protein were separated by 4-12% sodium dodecyl sulfate-polyacrylamide (SDS-PAGE) gel electrophoresis (Beyotime Institute of Biotechnology, Jiangsu, China) according to molecular weight. Then, the proteins were electrically transferred onto a piece of polyvinylidene fluoride (PVDF) membrane (Millipore, Bedford, MA, USA). After being blocked by nonfat milk in TBST, PDVF membranes containing proteins were incubated with indicated primary antibodies: anti-E-cadherin,1 : 5000; anti-N-cadherin, 1 : 5000; anti-Keap-1, 1 : 2000 dilution; anti-Nrf2, 1 : 2000 dilution; anti-HO-1, 1 : 1000 dilution; and anti-GAPDH, 1 : 1000 dilution, 4°C overnight. Next, the membrane was incubated with horseradish peroxidase-conjugated anti-rabbit IgG secondary antibody, 1 : 5000, 1 h at room temperature. Ultimately, the protein bands were detected using western enhanced chemiluminescence (ECL) substrate (Share-bio, Shanghai, China). GAPDH was selected to be the loading controls.

### 2.7. Construction and Selection of HO-1-shRNA Lentiviral Expression Vector

To knock down HO-1 (GenBank human, Gene ID:NM_002133), shRNAs targeting HO-1 were synthesized by Invitrogen (Beijing, China). We constructed HO-1-shRNA lentivirus expression vectors including shHO-1-1#, shHO-1-2#, and shHO-1-3#, and the optimal one was screened by real-time PCR and western blot. Primer sequences are listed in Table 1.

### 2.8. Real Time-Polymerase Chain Reaction (RT-PCR)

Total cellular RNA was isolated using TRIzol reagent according to the manufacturer's protocol (Invitrogen; Thermo Fisher Scientific, Inc). The cDNA was synthesized from total RNA using the PrimeScript 1st Strand cDNA Synthesis Kit (Takara Biotechnology Co., Ltd., Dalian, China). RT-PCR was performed using the SYBR Premix Ex Taq II (TaKaRa, Kusatsu, Japan). The relative mRNA expression of HO-1 was normalized by GAPDH. The primers of HO-1 and GAPDH were purchased from Sangon (Shanghai, China), and the primer sequences are listed as follows: (F: forward; R: reverse) HO-1, F: 5′-GGCCTCCCTGTACCACATCT-3′, R: 5′-CTGCATGGCTGGTGTGTAGG-3′; GAPDH, F: 5′-CAGGAGGCATTGCTGATGAT-3′, R: 5′-GAAGGCTGGGGCTCATTT-3′. Data represents the mean value ± SD from at least three independent experiments.

### 2.9. Xenograft Mouse Experiment

The animal experiment was carried out in accordance with relevant guidelines and regulations approved by the Animal Care and Use Medical Ethical Committee of School and Hospital of Stomatology, Shandong University. 12 Male BALB/c nude mice (6 weeks of age) purchased from the National Laboratory Animal Center were randomly divided into 2 groups, with 6 mice in each group. CAL27 cells (2 × 10^7^ cells per injection) were subcutaneously injected on the right groin of each mouse. After transplantation for 14 days, each group of mice received an intraperitoneal injection of PBS (control group) or 30 mg/kg CORM-3 every other day for 3 weeks. The size of the subcutaneous tumor in nude mice was measured every 3 days. Tumor volume was measured by a caliper and calculated using the following equation: *V* = *π*/6 × *L* × *W* × *W* (L = length, *W* = width).

### 2.10. Immunohistochemistry (IHC)

Animals were killed five weeks later after implantation, and the tumors were detached and weighed immediately. Half of the tumor tissues were fixed with 4% paraformaldehyde (PFA), embedded in paraffin, and sliced into 5 *μ*m thick sections for IHC staining. The sections were then deparaffinized in xylene and rehydrated in graded ethanol washes. Endogenous peroxidase activity was quenched with 3% hydrogen peroxide for 15 min at room temperature, and then, the sections were boiled in citrate buffer at 121°C for 10 min to retrieve antigenicity. The sections were incubated with anti-Ki67, 1 : 200, and anti-HO-1, 1 : 100, 4°C overnight, followed by incubation with streptavidin-peroxidase conjugated secondary antibody for 25 min at 37°C, and then, DAB staining was performed. The images were captured under a light microscope (Olympus, Tokyo, Japan). The Image-Pro Plus 6.0 software (Media Cybernetics, Rockville, MD, USA) was used to obtain the integrated optical density (IOD) value of Ki67, E-cadherin, and HO-1 staining.

### 2.11. Statistical Analysis

SPSS software, version 23.0, was used to analyze data. Data were shown as the mean ± standard deviation (SD). Student's *t*-test or one-way ANOVA followed by the least square difference (LSD) was performed for comparisons. *P* value < 0.05 was considered statistically significant.

## 3. Results

### 3.1. CORM-3 Inhibits Proliferation of TSCC Cells

In order to investigate the effect of CORM-3 on CAL27 and SCC4 cell proliferation, CAL27 or SCC4 cells were stimulated with CORM-3 at concentration of 0, 100, 200, 400, and 800 *μ*M, respectively, for 24 h. Cell proliferation was detected by CCK-8. The results showed that the proliferation of CAL27 and SCC cells was significantly inhibited by CORM-3 at 400 and 800 *μ*M concentrations (Figure 1(a)). We further studied the effects of different concentrations of CORM-3 and different treatment times on the proliferation of TSCC cells (Figures 1(b) and 1(c)). CAL27 and SCC4 cells were stimulated with CORM-3 at 0, 200, 400, and 800 *μ*M, respectively, and cell proliferation was measured at 6, 12, 24, 48, and 72 h after treatment using CCK-8 assay. As the dose increased, the inhibitory effect of CORM-3 became more potent, and the proliferation of the CAL27 and SCC4 cells was inhibited in the concentration of 400 *μ*M at 24 h and then entered the plateau stage after 48 h, which verified the time and dose dependence of the inhibitory effect of CORM-3 on cell proliferation. CORM-3 at the concentration of 400 *μ*M was the lowest inhibitory concentration for inhibiting cell proliferation, indicating the 400 *μ*M was the optimal dose of CORM-3.

Subsequently, CAL27 and SCC4 cells were treated with 400 *μ*M CORM-3, iCORM-3, and negative control medium for 24 h. CCK8 showed that the proliferation of cells was significantly inhibited by CORM-3, whereas there was no difference between the iCORM-3 and the control group (Figure 1(d)).

### 3.2. CORM-3 Inhibits Migration and Invasion of TSCC Cells

Scratch assays were implemented to explore the effect of CORM-3 on TSCC cell migration. The CAL27 or SCC4 cells were cultured in the presence of CORM-3 (400 *μ*M). For both cell lines, iCORM-3 treatment or normal medium resulted in early 100% of the wound close after 24 h. However, CORM-3 treatment retarded the wound close, as shown in Figures 2(a) and 2(b). Quantitative analysis showed that the migration of CAL27 and SCC4 cells treated with CORM-3 was significantly lower than that of cells in iCORM-3 or NC group at 6 h, 12 h, and 24 h. Transwell chamber was used to investigate the potential effect of CORM-3 on the invasion of CAL27 or SCC4 cells. We found that the invasion capacities of CAL27 and SCC4 cells treated with CORM-3 declined almost 60% compared with that in iCORM-3 or the control group (Figures 2(c) and 2(d)). These results suggested that CORM-3 significantly inhibited the migration and invasion of TSCC cells.

In order to explore the mechanism underlying the regulatory effect of CORM-3 on the migration and invasion of TSCC cells, we checked the expression of the factors E-cadherin and N-cadherin, which were related to cell migration and invasion.

As shown in Figures 2(e) and 2(f), the protein expression level of E-cadherin in CAL27 and SCC4 cells treated with CORM-3 was significantly increased, while the N-cadherin expression was decreased. These results indicate that CORM-3 may inhibit the EMT of TSCC cells, thereby inhibiting the migration and invasion of TSCC.

### 3.3. CORM-3 Regulated the Keap1/Nrf2/HO-1 Pathway

Cells were treated with 0, 100, 200, and 400 *μ*M CORM-3 for 24 h, and then 400 *μ*M CORM-3 stimulated cells at 0, 0.25, 0.5, 1, 3, 6, and 12 h, respectively, and total protein was extracted. Western blot was used to detect the effect of CORM-3 on HO-1 protein expression in CAL27 and SCC4 cells. The results showed that the expression of HO-1 upregulated with the increased concentration of CORM-3 (Figures 3(a) and 3(b)). Moreover, HO-1 expression increased gradually at 0.25, 0.5, 1, 3, 6, and 12 h in CAL27 and SCC4 cells (Figures 3(c) and 3(d)).

To confirm whether CORM-3 exerted its function through the HO-1 pathway in TSCC cells, we constructed a HO-1-specific shRNA to knock out its expression. Efficacy was confirmed by RT-qPCR and western blot (Figures 3(e) and 3(f)). Next, we further conducted the rescue assays through a series of biological behavior experiment. As shown in Figures 3(g) and 3(h), compared with the NC group, the proliferation of CAL27 and SCC4 cells in the shHO-1 group was significantly promoted. However, knockdown of HO-1 could partially abrogate the inhibitory effect of CORM-3 on the proliferation of TSCC cells.

We also performed wound-healing and transwell assay after HO-1 knockdown. In the migration assay, we found that the migratory capacities were reversed in the shHO-1-treated CAL27 and SCC4 cells compared with those in the CORM-3 group (Figures 3(i) and 3(j)). Similarly, the invasive capacities of CAL27 and SCC4 cells were increased by 50% in the shHO-1 group (Figures 3(k) and 3(l)).

Studies have shown that the Keap1/Nrf2/HO-1 antioxidative stress signaling pathway play vital roles in cell migration [21]. Therefore, we detected the expression levels of Keap1 and Nrf2 at 0, 0.25, 0.5, 1, 3, 6, and 12 h after CORM-3 treatment in CAL27 and SCC4 cells by western blot. We found that the expression of Keap1 was downregulated and the expression of Nrf2 was upregulated with the increase of CORM-3 treatment time (Figures 3(m) and 3(n)).

The above results suggested that CORM-3 treatment of TSCC cells can activate the Keap1-Nrf2-HO-1 signaling pathway, and the effect was time-dependent.

### 3.4. CORM-3 Inhibits Tumor Growth *In Vivo*

To evaluate the role of CORM-3 on TSCC in vivo, we used a xenograft mouse model. CAL27 cells were subcutaneously injected into the left armpit of nude mice. At 2 weeks, the tumor-bearing mice were injected with CORM-3 (30 mg/kg) or PBS every other day, and then, the effect of CORM-3 on the growth of subcutaneous tumors in nude mice was observed. Up to 14 days after treatment, the growth volume of subcutaneous tongue squamous cell carcinoma in mice injected with CORM-3 intraperitoneally was significantly smaller than that of the control group (Figures 4(a)–4(d)). Moreover, immunohistochemical analysis of xenograft tumors confirmed that the proliferation marker Ki67-positive cell in the tumor tissue of the CORM-3-treated group was significantly lower than that in the control group, and protein HO-1 expression increased significantly in comparison with the control group (Figure 4(e)). Similarly, the protein expression of HO-1 in tumor tissue of nude mice was significantly lower than that in the control group (Figure 4(f)). These results above supported our *in vitro* findings and indicated that CORM-3 inhibited the growth of TSCC cells *in vivo*.

## 4. Discussion

CO has long been considered a freely diffusible and toxic gas molecule because its binding affinity is 400 times that of oxygen, which can lead to CO poisoning and eventually respiratory failure. However, recent research shows that CO can act as an intracellular messenger molecule with multiple biological functions, including anti-inflammatory, antioxidant, and anticancer [22, 23]. CORMs are effective in regulating CO release *in vivo* and *in vitro* at appropriate circumstances [24]. The basis of CORM as a therapeutic agent is to deliver a controlled amount of CO to tissues and organs. CORM-3 was found to inhibit the expression of inflammatory cytokines COX-2, PGE2, and RANKL in human periodontal ligament stem cells (hPDLSCs) induced by LPS and nicotine, and the anti-inflammatory effect was mediated by the HO-1 signaling pathway [25]. It has been confirmed that CORM-3 could inhibit osteoclast differentiation and maturation through the HO-1 pathway in osteoclastogenic differentiation of RAW264.7 cell [26]. CORM-3 could also promote the osteogenic differentiation of BMSCs and significantly increase the expression of HO-1 [27]. Recent studies have shown that CORM-3 could activate Nrf2 by inducing HO-1 expression in rat brain astrocytes [28]. In our study, we used CAL27 and SCC4 cells to investigate the effects of CORM-3 on TSCC cells and explored the underlying mechanism of CORM-3. The research showed that CORM-3 not only inhibited the proliferation, migration, and invasion of CAL27 and SCC4 cells *in vitro* but also inhibited tumor growth *in vivo*. We observed that the growth of TSCC xenograft on mice was inhibited by the treatment of CORM-3. The expression level of Ki67 in tumors was downregulated, while the HO-1 expression was upregulated. We also analyzed the expression of several molecules related to the biological function of CORM-3 on TSCC cells. Treatment of CORM-3 could affect the protein expression of the migration- and invasion-related EMT markers E-cadherin and N-cadherin in a time-dependent manner. We also detected the effect of CORM-3 on HO-1 protein expression in CAL27 and SCC4 cells and found that the expression of HO-1 upregulated with the increased concentration of CORM-3 and was time-dependent. In order to prove these effects, we inhibited the HO-1 expression by sh-RNA and performed the same experiment. Results showed that knockdown of HO-1 could partly restore the inhibitory effect of CORM-3 on TSCC cells, indicating that this inhibitory effect was mediated partially by HO-1.

EMT is associated with functional changes related to metastasis, i.e., enhanced migration and invasion. EMT is a process of phenotypic change from epithelial to mesenchymal, accompanied by high expression of N-cadherin and Vimentin, while low expression of E-cadherin [29]. NF-E2-related factor 2 (Nrf2) is the main regulator of cells in response to environmental stress and the main regulator of many cytoprotective genes [30]. Nrf2 has been confirmed to promote the EMT process in various cancer cells. Feng et al. [31] reported that macrophage Nrf2 activation can induce EMT process in hepatocellular carcinoma. In addition, Nrf2 facilitated the migration of breast cancer cells by affecting the EMT expression [32]. Keap1 is a sensor for oxidative stress and specifically targets the Nrf2 [33, 34]. Keap1 and Nrf2 form trimers, which accelerate the ubiquitination of lysine residues in Nrf2 neh2 domain, leading to the proteasome degradation of Nrf2 [35]. The Keap1/Nrf2 pathway is essential for protecting the cells against stress. miR-200a inhibits oxidative stress and inflammatory response by suppressing Keap1 and activating the Nrf2 pathway in the development of liver disease [36]. HO-1, a member of the heme oxygenase family, has anti-inflammation, antioxidation, and regulating angiogenesis effects, and it is regulated by Nrf2 [37]. Many studies have shown that activating the common oxidative stress pathway Keap1-Nrf2-HO-1 can rescue cells with oxidative damage [38]. However, HO-1 may play an anticancer effect in a variety of cancers, such as prostate cancer, breast cancer, non-small-cell lung cancer, and pancreatic cancer. Overexpression of HO-1 or treatment of non-small-cell lung cancer cells with CO-releasing molecule-2 can downregulate the expression of miR-378, inhibit the expression and synthesis of angiogenesis-related factors, and then play an antitumor effect [17]. In our study, we detected the expression of Keap1, Nrf2, and HO-1 and found that the expression of Nrf2 and HO-1 was increased while Keap1 was reduced in TSCC cells with the treatment of CORM-3. In summary, we can conclude that CORM-3 can suppress TSCC cell proliferation, migration, and invasion which is regulated by the EMT process and mediated by the Keap1/Nrf2/HO-1 signaling pathway.

Importantly, for the first time, our results indicated that CORM-3 can inhibit the expression of Keap1 protein to relieve the inhibition of Nrf2 activity by Keap1 protein, thereby promoting the HO-1 protein expression in TSCC cells. The deficiency of our study is that a group of chemotherapeutic drugs was not reserved as a positive control in animal experiments to compare the differences, advantages, and disadvantages of CORM-3. In addition, pharmacokinetics and toxicology of the antitumor effect of CORM-3 are still insufficient, which need to be verified in subsequent experiments.

In conclusion, our findings demonstrated the inhibitory effect of CORM-3 on proliferation, invasion, and metastasis in TSCC cells. CORM-3 regulates the biological functions of TSCC cells by regulating the EMT process. Additionally, CORM-3 exhibits a tumor suppressor effect on TSCC by activating the Keap1/Nrf2/HO-1 antioxidant pathway. Our findings may reveal a new potential therapeutic strategy for TSCC treatment.

## Figures and Tables

**Figure 1:** The effect of CORM-3 on TSCC cell proliferation. (a) CAL27 or SCC4 cells were incubated with 0, 100, 200, 400, and 800 *μ*M CORM-3, respectively, for 24 h. Cell proliferation was assessed by a CCK-8 kit. (b, c) CORM-3 of 0, 200, 400, and 800 *μ*M was applied to CAL27 and SCC4 cells, respectively. Cell proliferation was measured at 6, 12, 24, 48, and 72 h after treatment with CCK-8. (d) CAL27 or SCC4 cells were incubated with 400 *μ*M CORM-3 and iCORM-3 for 24 h. ^∗^*P* < 0.05 and ^∗∗∗^*P* < 0.001 vs. the control group, respectively.

**Figure 2:** The effect of CORM-3 on TSCC cell migration and invasion. (a, b) The effect of CORM-3 on the migration of CAL27 and SCC4 cells was tested using scratch assay (magnification, ×40). Statistical analysis of the healing distance showed that CORM-3 treatment could migrate at a lower rate than that in control group and iCORM-3 group. (c, d) The effect of CORM-3 on the invasion of CAL27 cells and SCC4 was tested by transwell assay (magnification, ×200). Cell numbers that invaded the lower membrane surface were less in CORM-3 stimulation groups than in the control group and iCORM-3 group. (e, f) Epithelial mesenchymal transition is involved in the CAL27 and SCC4 cells by CORM-3. CAL27 and SCC4cells were treated with CORM-3 for 0, 0.25, 0.5, 1, 3, 6, and 12 h; the protein expression of E-cadherin and N-cadherin was assessed by western blotting. Relative protein level was normalized to the corresponding GAPDH protein expression. ^∗^*P* < 0.05, ^∗∗^*P* < 0.01, and ^∗∗∗^*P* < 0.001 vs. the control group, respectively.

**Figure 3:** The regulatory effect of CORM-3 on the Keap1/Nrf2/HO-1 signaling pathway in the CAL27 and SCC4 cells. (a, b) CAL27 and SCC4 cells were treated with 0, 100, 200, and 400 *μ*M CORM-3 for 24 h, and western blot was used to detect the protein expression of HO-1. (c, d) CORM-3(400 *μ*M) stimulated cells at 0, 0.25, 0.5, 1, 3, 6, and 12 h, respectively. Western blot was used to detect the effect of CORM-3 on HO-1 protein expression. (e) The efficacy of HO-1specific shRNA was measured by RT-qPCR. We finally chose sh-HO-1-3# as the interference sequence. (f) The efficacy of shHO-1-3# was measured by western blot. (g, h) The effect of shHO-1 on the inhibitory effect of CORM-3 on the proliferation of CAL27 and SCC4 cells. Cell proliferation was assessed by a CCK-8 kit. (i, j) The effect of shHO-1 on the inhibitory effect of CORM-3 on the migration of CAL27 and SCC4 cells. Quantification of relative migrating distances of cells with indicated treatment. (k, l) The effect of shHO-1 on the inhibitory effect of CORM-3 on the invasion of CAL27 and SCC4 cells. Quantification of the invaded cells with indicated treatment. (m, n) CAL27 and SCC4 cells were treated with CORM-3 for 0, 0.25, 0.5, 1, 3, 6, and 12 h, and the protein expression of Keap1 and Nrf2 was assessed by western blotting. Relative protein level was normalized to the corresponding GAPDH protein expression. ^∗^*P* < 0.05, ^∗∗^*P* < 0.01, and ^∗∗∗^*P* < 0.001 vs. the control group, respectively. ^*P* < 0.05 and ^^*P* < 0.01 vs. comparison between two groups.

**Figure 4:** The effect of CORM-3 on the subcutaneous tumor growth of CAL27 cells in nude mice. (a) Images of the mice. (b) The body weights of the mice were measured twice a week for 5 weeks. (c) Images of the tumor specimens. (d) Tumor volumes were measured twice a week for 5 weeks. (e) The expression of Ki67 and HO-1 in the tumors was detected by immunohistochemistry staining. The IOD of Ki67 and HO-1 staining was quantitatively analyzed using Image-Pro Plus 6.0 software. (f) The protein expression of HO-1was detected by western blot in the tumors of nude mice. ^∗^*P* < 0.05 vs. the control group (*n* = 6).

**Table 1:** Primer sequences of shHO-1.

Genes	Forward (5′→3′)	Reverse (5′→3′)
shNC	CCGGCCTAAGGTTAAGTCGCCCTCGCTCGAGCGAGGGCGACTTAACCTTAGGTTTTTG	AATTCAAAAACCTAAGGTTAAGTCGCCCTCGCTCGAGCGAGGGCGACTTAACCTTAGG
shHO-1-1#	CCGGCCCTGTACCACATCTATGTTTCTCGAGTTGGGACATGGTGTAGATACATTTTTG	AATTCAAAAACCCTGTACCACATCTATGTTTCTCGAGTTGGGACATGGTGTAGATACA
shHO-1-2#	CCGGCAGCAACAAAGTGCAAGATTTCTCGAGTTGTCGTTGTTTCACGTTCTATTTTTG	AATTCAAAAACAGCAACAAAGTGCAAGATTTCTCGAGTTGTCGTTGTTTCACGTTCTA
shHO-1-3#	CCGGCCAGCAACAAAGTGCAAGATTCTCGAGTTGGTCGTTGTTTCACGTTCTTTTTTG	AATTCAAAAACCAGCAACAAAGTGCAAGATTCTCGAGTTGGTCGTTGTTTCACGTTC

## Data Availability

All data are available. Please contact the first author or the corresponding author.

## Abbreviations

CO: Carbon monoxide
CORM-3: Carbon monoxide-releasing molecules-3
iCORM-3: Inactive carbon monoxide releasing molecule-3
TSCC: Tongue squamous cell carcinoma
HO-1: Heme oxygenase-1
EMT: Epithelial mesenchymal transition
CCK-8: Cell Counting Kit-8
FBS: Fetal bovine serum
Nrf2: Nuclear factor, erythroid 2 like 2
Keap1: Kelch-like ECH-associated protein 1.
